# Complex young lives: a collective qualitative case study analysis of young fatherhood and breastfeeding

**DOI:** 10.1186/s13006-016-0066-9

**Published:** 2016-04-02

**Authors:** Jennifer Ayton, Emily Hansen

**Affiliations:** University of Tasmania School of Social Science, Hobart, Tasmania Australia; Menzies Institute for Medical Research, Tasmania, School of Social Science, Hobart, Tasmania Australia

**Keywords:** Breastfeeding, Young fatherhood, Socioeconomic disadvantage

## Abstract

**Background:**

Of all births in Australia, 10 % are to young fathers aged less than 24 years. How young fathers experience any breastfeeding and how this is shaped by their social context is poorly understood. Our aim is to increase understanding of the lived experience of young fathers (aged less than 24 years) and to explore the way they speak about breastfeeding in the context of their lives and parenting.

**Methods:**

This collective case study analysis uses qualitative data from interviews and focus groups with young fathers (aged less than 24 years) and community support staff. The research was undertaken in Tasmania, Australia, March to December 2013.

**Results:**

Young fathers in our study had complex social and emotional circumstances that meant breastfeeding was not a high priority despite them valuing the health benefits of breastfeeding for their babies. If supported by peers and their community they appear to have a more positive parenting experience.

**Conclusion:**

Breastfeeding although understood by the young fathers in our study as healthy and desirable is not a priority in their lives. Learning to be a parent and support their partners to breastfeed may be more effectively gained through mentoring and father-to-father localized community based support services.

## Background

Early parenthood (<24 years) makes up a small but significant proportion of all births in Australia [1]. Ten precent are to fathers aged < 24 years and 17 % are to young mothers aged < 24 years, with 6.1 infants born per 1000 teenage women aged < 19 years in 2012 [1].

Age is an important determining factor of breastfeeding practices. Young mothers either do not elect or continue to breastfeed [2]. Those who do commence have an 11 % increased risk of stopping exclusive breastfeeding (where the infant is fed only breastmilk) within the first six months [3]. Compared to young mothers, little is known about young father’s perceptions of breastfeeding. The dominant understanding how young mothers experience breastfeeding is often indirectly extended to young fathers [4] and the mother’s views are often taken as a proxy measure for the young fathers’ attitudes about breastfeeding [5]. From this perspective young fathers are assumed to be disengaged and to just ‘go along’ with the mother’s infant feeding choice. As a result of becoming a young father, men often experience the same level of social exclusion, stunted education, and job insecurity as reported for young mothers [6].

Early fatherhood is challenging and like young mothers, men may suffer from anxiety, depression, family isolation and rejection [7]. However young men are less likely to report it or seek help [8]. Despite this for some young men and their partners becoming a young parent is normal in their social context, offering them social status and emotional, sometimes educational and social support networks that would be unavailable to them in the mainstream setting [9, 10]. Thus young parenthood can offer advantages.

How young fathers experience any breastfeeding is poorly understood. Very little has been written about their views, despite growing recognition of the importance of fathers’ views on mothers’ breastfeeding practices [3, 4].

To address this gap we report on the young fathers’ experiences, and the views of professional community support staff (social workers, community nurses and teachers) who work closely with young parents to explore how young fathers experience breastfeeding and how the process of feeding infants is undertaken within the young fathers’ lives.

## Methods

We use a collective case study approach [11] to explore the complex nature of young fatherhood < 24 years, and breastfeeding (where the infant receives breastmilk, expressed or from a wet nurse, and any other food or fluids) [12], using a variety of qualitative data sources; semi structured interviews, focus group (FG) and field notes. Case study analysis is a valid tool for exploring complex phenomena and reveals deeper understandings of the lived experiences because it draws from collective sources [11].

The collective data sources are derived from a larger qualitative study undertaken from March to December 2013, in Southern Tasmania that explored the role of fathers in supporting breastfeeding. Ethics approval was granted though the University Tasmania Human Research Ethics Committee [H0011838]. This larger study used purposeful sampling to achieve a sample of 51 participants, including 37 parents (26 fathers and 11 mothers’) with infants/children aged less than 24 months, 11 professional community support staff (CSS) (social workers, community health nurses, secondary school teachers) whose roles included the coordination of community based parenting programs, counseling and outreach support for parents and who were living in Tasmania. Participants consented to and were offered either one to one semi structured interviews (phone or in person), or a focus group for those who were more comfortable talking as a group. All interviews and focus groups were audio taped, and transcribed verbatim. Observational and some interview data were collected as field notes. All participants were given pseudonyms to preserve confidentially.

A subset of data from this larger study were used to form the collective case analysis [11]. This included data from five young fathers (<24 years): one semi structured face to face interview; one FG involving four young men all of whom were living in socioeconomically disadvantaged areas of Tasmania, five one to one interviews with five professional CSS (three male and two female), reflections and field notes.

The data were analysed using iterative thematic analysis. Both JA and EH independently coded relevant FG, interview transcripts and field notes first, progressing to meeting regularly to develop thematic categories and form a consensus [13]. We focused our analysis using the following aim: to increase understanding of the lived experiences of young fathers aged < 24 years and to explore the way they speak about breastfeeding in the context of their lives. Thematic categories were developed and then subsumed into two overarching categories: ‘complex experiences’ and ‘talking about breastfeeding: no one ever asked’ [11].

## Results

The results are constructed within the context of young fatherhood and weave together excerpts from field notes and transcripts with the CSS and young fathers, describing firstly the experience of young fatherhood followed by how breastfeeding was talked about.

### The context of young fatherhood: ‘It’s really hard you know’

It was clear that the young fatherhood posed many challenges for fathers and CSS. Young men often spoke of how they struggled with ‘lots of stuff lot of problems’ (Ben 19 years Interview), including negotiating foster care, schooling and finding employment, the lack of information and support. Fathers often described feeling confronted, confused and isolated by early parenthood, explaining that they did not know what to do, where to go for help and or who to trust. Peter a CSS reflected that ‘if you're 16 and had a pretty rough trot in life and you're suddenly thrust into fatherhood, man, you've got no hope, or very limited hope really’. Other CSS empathetically spoke about young men ‘not wanting to be fathers,’ of ‘being scared’ and ‘not being mature enough to understand what it meant to be a father’. (Richard & Sarah. CSS) According to Richard this was because the young fathers lacked role models. The following quote from Peter a CSS summarizes the reality for the young father:

The young dad is challenged by the containment of parenting, they're used to mates, Play-station, that sort of stuff, getting out and about, and suddenly there's this responsibility there. We have had some tremendous successes with young dads, 18-year olds, either through reunification with child protection or through our family support programs where they've stepped up to be the parent where the child might have been removed from the mum, and yeah they've done a good job. That acceptance stage of oh yes I am a dad therefore I need to be responsible and therefore I need to learn. They rarely ever come forward on their own behalf wanting to learn how to be a good parent, they don't actually realise I don't think that these are these parental thoughts and ideas you have to have.

From the conversations during dedicated father-to-father and family support programs that Peter referred to in the above quote were limited or felt to be inappropriate for young fathers. Interviews with CCS revealed concerns over a perceived ‘gap’ in services, and how young men were generally unaware of where to access support or information citing ‘there is nothing for the young fathers especially those still at school’. (Michael) Traditional support avenues such as mothers groups were referred to as ‘no go zones’. Peter (CSS) explained that ‘men generally are excluded from parenting services because they are aimed at mothers’. Similarly Paul a father of three lamented ‘I’m not welcome at mothers groups’. (Paul, 22 years FG) The lack of dedicated father focused support services appeared to exacerbate feelings of personal isolation. Young men frequently expressed how they were unaware of the existence of dads groups before their infants were born. CSS staff empathized that preventative action was required stating ‘I think the best thing we can do is put more emphasis on education. Educating people before the event. I think after the event [birth] it’s really hard. It’s REALLY hard’. (Michael, CSS).

For the most part the young fathers appeared to gather support and information about parenting and feeding from peers or from their partners’. The four young men who took part in the focus group where all aged 21–23 years, lived in the same suburb. For them young parenthood was not disruptive or viewed as a ‘huge problem,’ Chris (23 years) explained; ‘it’s okay, not big deal, we all have young kids’. For these young fathers early parenthood increased social connectivity, and was viewed as ‘normal’ for young men to have young kids. All were living with the mothers of their children, had their children full time, were employed, ‘most of the time’ and had talked of social supports. However Dave (father of three) who was 18 years when he first became a father recalled how difficult being a young parent was and spoke of the stress and confusion of being a first time young dad ‘I was out of control, SO hard’. He talked of needing his partner to help him ‘get through it’ and of how much he enjoyed being a dad now; ‘there’s nothin’ better’. (Dave, 21 years FG).

The social connectivity of young fatherhood appeared to generate strength and help the young men adapt to the demands of parenting. Together the four young men spoke freely about how they relied on each other when resolving parenting and feeding problems. They socialised and shared food together, often advising each other on how to manage children who experienced bad dreams, how to feed their kids wild wallaby ‘even though the wife don’t like it,’ how much formula cost and where to get ‘cheap milk’ and or the cheapest food. For these young men fatherhood was clearly used as a mechanism to group together and to support each other.

### Talking about breastfeeding: no one ever asked

The young fathers confided that they had never shared their stories about breastfeeding with anyone. This was because as Paul (22 years) explained they ‘never thought about it before,’ exclaiming that ‘no one ever asked’. All of the young fathers regardless of how they feed their infants, considered breastfeeding as normal and best, ‘it’s best for the kid’. (Ben 19 years. Interview) Chris (23 years) from the FG reinforced this saying ‘it’s good…I think it’s good for the kid if the mum can do it’.

However, despite their positive views on breastfeeding, their partners had all stopped breastfeeding due to ‘problems.’ Chris recalled ‘she [partner] just had so many problems and everyone telling us something different’. It was clear that the fathers recognised similarities in each other’s and their partners’ breastfeeding experiences, with all reporting ‘we wanted to’ and that their infants had commenced at birth and then stopped breastfeeding within the first weeks after birth; exclaiming ‘my baby didn’t grow,’ ‘she [partner] had lots of pain,’ ‘the milk dried up’ or ‘she just couldn’t do it’. (Young fathers FG).

Early hospital breastfeeding experiences played an important part in how the fathers viewed their own personal breastfeeding experience. All young fathers talked about feeling ‘a little left out’ and how their partners received conflicting professional advice. This negatively impacted on their partners’ confidence and consequently the fathers who frequently expressed concern for their infants and partners. From the conversations, clearly health professionals were interpreted as supporting and encouraging. Paul (22 yrs) from the FG explained ‘I know they were just trying to help’ but the mixed messages ‘everyone saying something different’, appeared to create confusion in complexity.

Both CSS and the young men felt on many occasions that health professionals had not listened to or trusted them because they were ‘young parents’. The young fathers interpreted the ‘barrage of advice on breastfeeding’ in hospital and in the first few weeks after birth as being ‘pushed to breastfeed’. (Sarah. CCS) When asked what would help the young fathers reproved ‘listen to the parents’. Three of the young fathers from the FG shared their experience in the following excerpt:

Yeah-different people [hospital staff] saying three different things ‘You know, ‘Do this. Do this. Do this. You’ve got to keep breastfeeding’ you know and they just won’t listen to what the parents are trying to tell them and not think, they just need to come to this sort of thing [Dads focus group], you know…(Dave, 23 years)

Listen to the parents. (Chris, 23 years)

Listen to the parents and you know, just give them a bit of reality check really [All of the fathers talking together]. (Paul, 22 years)

Peter (CSS) sentiments conclude the fathers’ experiences aptly; ‘so that's a clear message time and time again, so whatever’s happening in there [hospital] it's not coming through well’.

The message that did appear to get through to the fathers was that breastfeeding is best for the child, but ‘formula is okay if you have to’. (Paul, 22 years) Despite breastfeeding being accepted as ‘best’ by the CSS and the young fathers, the staff pondered that in the context of their often chaotic and challenging lives ‘breastfeeding was well, it’s not a big thing breastfeeding, it’s just not a priory for them’. (Anne and Michael. CSS) The fathers in the FG reiterated this; it [breastfeeding] was just too hard, she was gutted when she stopped’. (Chris, 23 years) Breastfeeding in the scheme of being as Peter (CSS) was quoted earlier ‘thrust into fatherhood’, job, income and housing insecurity, going to school, family tension, and foster care obligations did not appear to be the focus despite the young agreeing that its good to do if you can.

One of the main threads running through the young men’s stories were the health benefits of breastfeeding for infants. Fathers were less aware of benefits for mothers and were familiar with the idea that breastfeeding is ‘natural’ and ‘good’ for infants. Ben (19 years) shared this view [breastfeeding as natural] and talked openly about what he described as the simplicity of breastfeeding when his partner breastfeed their infants. He reminisced about when the ‘littlie’ had come home from hospital and the family was together as unit. Breastfeeding ‘it’s expected’ he shrugged his shoulders to acknowledge that ‘it’s just what you do’. ‘Yeah good [breastfeeding] it’s easier and better for them, it’s meant to be full of good things for the kid’. He went on to recount his experience:

Yeah it is easier they wake up and she just flopped it out and feed the baby… a lot easier than getting up in the night to get a bottle. She was really dirty on it when the milk dried up and the littlie ended up on a bottle at 2 weeks. It hurt too I think [meaning the stopping hurt]. She [partner] was really bummed when she stopped.

Similarly the young fathers in the FG shared their breastfeeding experiences and agreed that it is ‘healthy and natural’. Dave explained how all of his children had started breastfeeding, sharing openly with his peers:

Well, Kate started breastfeeding, but my partner had the same problem with not getting enough milk for the baby which was great when they were breastfed because I’d sleep all night, but then once they went to bottles, my partner slept all night and I didn’t [Laughter from the group] Yeah but, I didn’t mind it. (Dave, 21 years)

How long did you breastfeed? (Interviewer)

Not for too long. Probably a few months, that was it. Because they just wasn’t growing like they should be so we just didn’t have much of a choice. In the end the Nurses would push at her to keep trying and keep trying, but when you see kids not growing like they should be, it’s like well we have to make this tough choice and…go with the bottle…so it would. (Dave)

And how was your partner? (Interviewer)

Really devastated. Yeah. It upset her quite a bit that she couldn’t keep breastfeeding and that we had to go to the bottle because she wanted to keep going. We just didn’t have a choice. (Dave)

So how was that for you? (Interviewer)

Oh well, it was hard but…I just had to help her along and make sure…the baby was fed. (Dave)

Were you sort of thinking it would be a better thing to go bottle? (Chris, 23 years)

Well I know the benefits of breastfeeding versus bottle feeding, but then there’s like they wasn’t putting on weight, like it was a health sort of thing that sort of had to push us into bottle feeding. We tried different things, changed her diet and got her eating all different things to try and help build up the flow, but it just wasn’t working at all, so we just had to do it. She got quite depressed over it and stuff like that, but we got through it. (Dave)

The young fathers were equally shocked and relieved to hear that others had experienced breastfeeding difficulties, Chris (23 years) exclaimed during the FG ‘thought it was only us’, this clearly caused them distress. All had hoped that their babies would be breastfed and were deeply disappointed for their partner when they ‘had to stopped breastfeeding’. They were also protective of their infants and partners and recognized the need to ‘feed the child’ so were happy to fit in and ‘to do whatever’ to make it work. Perceiving that they had ‘no control over what happened’ referring to ‘we just didn’t have a choice’. (Young Fathers FG)

## Discussion

This paper contributes to the understanding of how breastfeeding is experienced in the context of young fathers’ lives and revealed two important insights. Firstly although considered important, breastfeeding is not a priority in the context of young fatherhood. This is despite the fathers finding some joy and viewing breastfeeding as the most ‘natural’ nutrition for babies. Contrary to the belief that young fathers and mothers have little interest in breastfeeding [2] fathers in this study highly valued breastfeeding and where often saddened by their partners stopping. The finding that the young fathers had not been asked or had ever thought to share their experiences about breastfeeding is alarming. It suggests that young fathers are often forgotten in the mother infant breastfeeding dyad, despite evidence showing that fathers feeding preferences have a significant influence of breastfeeding outcomes [3]. Other studies have also found that fathers across the social spectrum value breastfeeding but may feel isolated [14–16] and are reticent to access support. Clearly there is a need to proactively involve the young father prior and post birth to support their partners to breastfeed.

The complexity of young parenthood and the associated social, economic and emotional disadvantage [17, 18] can easily push breastfeeding into a ‘too hard basket’. Feeling pressure to breastfeed, confused by conflicting messages and observing their partners and infants struggle with breastfeeding generates stress, feelings of isolation and helplessness. This may contribute to and explain the young father feeling that breastfeeding is just too hard [15, 19]. For young fathers who are often struggling with complex social circumstances [20] negotiating breastfeeding and supporting their partners to breastfeed in the context of a myriad of other new and sometimes difficult changes is very challenging. Understanding these complexities may help health professionals to frame young parenthood and breastfeeding as a positive way to promote health and family bonding.

Early parenthood has often been considered damaging and leads to a trajectory of disadvantage and social isolation [17, 21]. Our study revealed that for some men early parenthood may offer a social network that as others have shown enriches their lives [10, 22]. Young men are often assumed to be disinterested and reluctant to become engaged with services or other fathers [23]. From our research whilst young fathers are not likely to come forward without prompting to seek information or support about breastfeeding or parenting, once supported they actively engage with the process [23]. If safe and trusted social networks in the form of peer namely father-to-father groups are established and young fathers are supported to attend, valuable mentoring is facilitated. Our findings support previous work showing this is particularly useful in the later teen years > 19 years [23], reproducing a positive effect on mother and child’s wellbeing, decreasing the social disadvantage associated with young and teenage parenthood [17, 21].

## Conclusion

Young fatherhood offered the young men in our study a social support network and a place in their communities. Although becoming a young father is experienced as hard and challenging, young men value breastfeeding and becoming a father. They approach breastfeeding with hope and wanting the best for their babies and aim to support their partners. Breastfeeding although understood by the fathers as healthy is not prioritized in their lives. For young men, developing the confidence and knowledge to parent and support their partners to breastfeed may be more effectively gained through mentoring and father-to-father localized community based support groups.
